# Designing an Optimum and Reduced Order Filter for Efficient ECG QRS Peak Detection and Classification of Arrhythmia Data

**DOI:** 10.1155/2021/6542290

**Published:** 2021-12-22

**Authors:** Hemant Amhia, A. K. Wadhwani

**Affiliations:** Electrical Engineering, MITS, Gwalior, MP, India

## Abstract

Electrocardiogram (ECG) is commonly used biological signals that show an important role in cardiac analysis. The interpretation and acquisition of QRS complex are significant measures of ECG data dispensation. The *R* wave has a vital character in the analysis of cardiac rhythm irregularities as well as in the determination of heart rate variability (HRV). This manuscript is proposed to design a new artificial-intelligence-based approach of QRS peak detection and classification of the ECG data. The design of reduced order IIR filter is proposed for the low pass smoothening of the ECG signal data. The min-max optimization is used for optimizing the filter coefficient to design the reduced order filter. In this research paper, elimination of baseline wondering and the power line interferences from the ECG signal is of main attention. The result presented that the accuracy is increased by around 13% over the basic Pan–Tompkins method and around 8% over the existing FIR-filter-based classification rules.

## 1. Introduction

It has been found by the World Health Organization that heart arrest is the world's most common cause for death [1]. Therefore, a strong focus has been put on cardiac health research with a focus on medicine, prevention, and technology which sequentially led investigators to work on educating cardiovascular skills that are usually applied in clinics and hospitals to make predictable diagnoses. Therefore, ECG signal analysis in the clinical heart test used to screen various heart defects is of prime importance. Digital signal processing has therefore been widely used to analyze the ECG signal over the past three decades.

Electrocardiogram (ECG) is an irregular signal that replicates cardiac activities. Most understanding of heart pathology is possible by studying ECG signal [1]. The evaluation matrix for healthy heart is heart rate and ECG signals. If we capture ECG signal from a patient and if there is any nonlinearity, then this is termed as cardiac arrhythmia [2].  Figure 1 shows a typical ECG beat.

The length and amplitude of the PQRS-TU wave have valuable evidence on the condition of the heart-related illness. The ECG signal aspects different varieties of noises during acquisition in the clinical field. The artifacts usually occurring are exterior electromagnetic field intrusion, noise from instruments, interference with the power line, clamor from electromyography (EMG), and noise from electrode connection. These artifacts influence frequency determination and signal superiority and have a strong effect on the morphology of the ECG data that contains essential cardiac foundations [3]. The problem of removing infected noises is recommended, which is important in the ECG data, and promotes accurateness.

ECG is a significant implementation for medical practitioners in the arena of cardiac health assessment and recognition. ECG is often adopted as a diagnostic approach for the detection of cardiovascular diseases by cardiologists [4]. The beginning of heart disease is extremely important because it can reduce sudden heart failure [5]. A high quality of ECG signals is required for precise diagnoses. Electrodes pasted on the body's skin are used to show and capture electrical heart activity [2, 3, 6]. The ECG signals include some of the following features: atrial depolarization of the P-wave component, the QRS complex designating ventricular depolarization, and a ventricular repolarization designated by *T* wave. Although the ECG signal is nonstationary in nature, a solid filters algorithm and well-known Hilbert transform can visually detect R-position peak's in order to derive analysis for the ECG data.

The R-peak finding work is carried out by the Hilbert transformation [6] using a cleaned ECG data taken out from the MIT-BIH arrhythmia database [5]. The suggested technique provides an improved measurement of accuracy, sensitivity, and predictivity in comparison of the previous results published.

Figure 1 represents the significant characteristics of an ECG wave whose significant features are P, *Q*, R, S, and *T*, and certain periods, such as P-R, S-T, and Q-T intervals, are shown in the typical scalar-electrocardiographic waveform. Healthy heart has regular rhythm which is also called a normal sinus rhythm (NSR). P-waves signify atrial depolarization [1]. The regular *Q* wave is an early descending deflection of the P wave and signifies septal depolarization. The R wave is the most usual waveform for the ECG to detect and characterize early ventricular depolarization. The S wave, which represents the late ventricular depolarization, is the first negative deflection after the *R* wave. The T-wave characterizes ventricular repolarization. U waves are a repolarization of the Purkinje fibres which show the latest ventricular residuals.

## 2. ECG Dataset

In order to implement this research in the MATLAB environment, a total of 18 ECG records have been adopted. The duration of each record is 30 minutes and 5556 seconds; the length below is rounded to the next second; due to accumulated rounding error, it cannot be exactly 30 : 06. Heart rates are measured over 3 R-R intervals in beats per minute [7].

## 3. Related Work

The papers on processing ECG data and QRS complex detection were developed by Peterkova et al. The QRS complex is detected using QRS online detector to determine the different peaks in the ECG using the state-owned logic, based on average and adaptive noise-and-signal thresholds [8]. Based on digital analysis of the pitch and amplitude, a real time algorithm was developed in this research article proposed by Jiapu Pan et al. to detect QRS complexes with ECG signals. The procedure inevitably regulates verges and parameters to adjust regularly for ECG fluctuations such as QRS morphology and heart proportion with increased detection sensitivity. 99.3% of the QRS complexes [9] are found in the accuracy of this algorithm.

Three methods for detecting QRS complex were implemented in a research paper projected by Vandana verma et al.; one is the adaptive threshold where the Pan–Tompkins Procedure was applied to identify the QRS complex. The Dynamic Quantized Threshold was another procedure. This method was used to eliminate entire frequencies, which is not essential to detect the section of the QRS complex by Butterworth filter having passing ensemble of 1–13 Hz. The mean was removed from the signal for the removal of the baseline. By quadrupling the signal, the gradient and moving average integrator detected four components. Finally, the preferred ultimate QRS feature was imitative by keeping the amplitude of G4 that is more than dynamic [10].

Using PNDM, Sameer K. Salih and coworkers were able to detect QRS complexes in ECG signals and evaluate related R-R intervals. Compared to other ECG signal waves, deflection QRS complexes occurring between R&S waves were found to have a large positive and negative interval. The proposed detection process followed a new fast direct algorithm applied to the ECG record itself, without any further transformations, such as the discrete wavelet transformation (DWT), or any filtering sequence [11]. According to Sharma et al., QRS complex can be detected using the synchrosqueezed wavelet transform (SSWT), which synchronizes with the wavelet's continuous transformation. The *R* peaks were detected using the nonlinear mapping technique [12].

Naaz et al. projected research work compacts with the extraction by wavelet decomposition of the QRS complex. The first preprocessed ECG signal was noisy for removing the walking mark and the base mark. The ST subdivision was also carried out to verify that the ECG model belongs or does not belong to patients with heart attack [13]. A paper proposed by Sivakumar et al. was used to represent the method of Empirical Mode Decomposition as arithmetic sum of zero mean AMFM constituents, in adaptive format. QRS complex detection was completed with EMD and combination of Haar wavelet transform to work better than other methods. The nonstationary signal such as ECG was directly applied to a notch filter with a ringing effect [14].

Yan sun et al. proposed a wave detection including QRS complex by using a transformation-based unique detector named multiscale morphological derivative [15].

Pan and Tompkins method [16] is used to calculate slope, amplitude, and width of ECG signal. After the preprocessing step, two sets of thresholds are applied to the signal to remove noise, smooth the waveform, and amplify the QRS slope and width to locate the true positive *R* peaks. In [17], which reproduced the same preprocessing phase, an evolution in the Pan and Tompkins procedure [16] is indicated. However, by performing performance tests on three estimators for the adaptive threshold (mean, median, and iterative maximum level), decision rules can be improved.

Using a robust algorithm, the Hilbert transformation is indicated in [18]. Using a Finite Impulse Response (FIR) filter window and Kaiser Bessel window, the ECG signal will be filtered to remove muscle artefacts and motion artefacts, as well as baseline noise. To determine the *R* peak, the first differential of the ECG signal is Hilbert.

The ECG database is stored in various cloud databases which can be accessed as per requirement [19–21] and these further discussed algorithms will be helpful to preprocess the ECG signal. The precisely cleaned ECG will support physiologists in the accurate detection of heart disease and accordingly the best possible treatment.

## 4. Problem and Challenges

The baseline wandering noise makes it difficult to analyze ECG data. For the correct evaluation of ECG, it is therefore necessary to suppress this noise. The basis of an ECG waveform can be significantly different. A variety of frequencies are diverted by both high and low amplitude. Before processing the ECG data, the major concern is therefore to remove the additive noise and the baseline noise.

A recorded signal is filtered, termed as online filtering. In the direction of examining the real time properties of stress on electrical heart activities, the signals are filtered and analyzed simultaneously.

An important research challenge is a reduced order filter for ECG processing hardware in real time. With the filter order reduced, the size of the filter over the hardware is lesser, but the accuracy of the ECG detection feature should not be decreased. The filter design coefficients can be optimized for this purpose. The algorithms applied for existing issues are discussed below.

### 4.1. Algorithms

There are many methods designed for improving the performance of ECG artifact removal in the front end processing. It is expected that peak detection and classification efficiency directly depends on the efficiency of methodology adopted at preprocessing stage. Thus in this paper two existing filtering strategies as Pan–Tompkins [17] and 60 order FIR filter are presented as shown in Algorithms 1 and 2, respectively.

The method of Pan and Tompkins is most widely used for the peak detection [17] as described in Algorithm 1. However, for improving the classification efficiency of ECG signal, many variants of Pan and Tompkins method were designed.  Algorithm 2 is the modified peak detection method using the 60 order FIR filter for preprocessing ECG for peak detection. In addition, this method also classifies the ECG as the regular or irregular heart.

## 5. Contribution of Work

This paper demonstrated the efficient use of optimization-based filter for ECG peak detection and classification. It contributes in the two passes. In the first pass, an efficient QRS peak detection algorithm is proposed using the designing of reduced order IIR filter using the transfer function optimization. The IIR filter is combined with Hilbert transform for performance improvement of peak detection. The filtering performance for baseline wondering is compared for three different approaches. In the second pass, the paper proposed a fuzzy ECG classification rule based on HRV parameters in time history analysis. The performance of the proposed rule is compared with two existing methods as Pan–Tompkins and FIR filter approach. The classification efficiency is compared based on true positives.

## 6. Proposed Methodology

The manuscript projected to design a new approach of QRS peak detection and classification in the ECG data using the reduced order IIR filter for the low pass smoothening of the ECG data. The optimization technique is proposed to minimize the order of the anticipated IIR filter design. The block illustration of the projected ECG classification method is presented in Figure 2.

The proposed IIR filter is a two-stage filter designed with the arrangement of the pass band and stop band filter as shown in Figure 3.

Let X(n) be the input ECG data to be filtered; then, the basic design of IIR filter in terms of transfer functions is defined as

(1) $$\begin{array}{c} Y\left(n\right)=X\left(n\right)*h_{1}*h_{2}, \end{array}$$

where *h*_1_ is the transfer function of the pass band filters; an example of transfer function for ECG data of 106 MIT-BIH is given as

(2) $$\begin{array}{c} h_{1}=\frac{\;0.2066\;s^{4}-0.4131\;s^{2}+\;0.2066}{s^{4}+\;0.5488\;s^{3}+0.4535\;s^{2}+\;0.1763\;s\;+\;0.1958}, \end{array}$$

where *h*_2_ is the transfer function of the stop band filter; an example of transfer function for ECG data of 106 MIT-BIH is given as

(3) $$\begin{array}{c} h_{2}=\frac{\begin{array}{c} 0.3201\;s^{16}+\;4.517\;s^{15}+\;30.45\;s^{14}+\;130\;s^{13}+\;393.2\;s^{12}+\;\\ 892.9\;s^{11}+1574\;s^{10}+2196\;s^{9}+2452\;s^{8}+2196\;s^{7}+1574\;s^{6}\\ +\;892.9\;s^{5}\;+393.2\;s^{4}+130\;s^{3}+30.45\;s^{2}+4.517\;s\;+\;0.3201 \end{array}}{\begin{array}{c} s^{16}+12.12\;s^{15}+70.25\;s^{14}+258.1\;s^{13}+672.2\;s^{12}\\ +1316\;s^{11}+2004\;s^{10}+2419\;s^{9}+2340\;s^{8}+1819\;s^{7}+113\;s^{6}\;\\ +559.4\;s^{5}+214.8\;s^{4}+62\;s^{3}+12.7\;s^{2}+1.649\;s\;+0.102 \end{array}}. \end{array}$$

Transfer function for IIR filter, pass band filter, and stop band filter is shown in equations (1), (2), and (3).

### 6.1. Methods

Most frequently applied ECG processing methods are discussed below.

#### 6.1.1. Pan and Tompkins (PT)

When Pan and Tompkins introduced the low-pass differentiation procedure (LPD) in 1985 [17], it revolutionized the ECG signal processing field. When detecting QRS, amplitude and width data applied algorithmic complexes in PT and the QRS finding [22] was not successful. There are three steps in the detection process. It is possible to create a digital system for the use of filtering, nonlinear transformations, and decision rules.

With the PT method, there is no significant power consumption. After being filtered with an analogue band-pass filter to limit the ECG signal's frequency range to about 50 Hz, the raw ECG signal is fed into an A/*D* converter, which digitizes the signal at about 200 Hz.

In order to perform pattern recognition, a band-pass filter is connected in sequence of low pass (LP) and high pass (HP) filter arrangement. To limit the ECG signal's operating range and to reduce higher frequency noise, a low pass filter (LPF) is used; whereas a high pass filter (HPF) highlights each QRS complex.

It is possible to process data in real time by using a digital filter with integer coefficients. All types of unwanted interferences and frequency noise impacts are greatly reduced by the overall band-pass filter. To identify and mark all of the R-peaks [23, 24], the ECG signal is conceded through a local peak recognition procedure. Using a set of thresholds, this algorithm selects the QRS complexes that are required. Adapting the threshold based on the peak's amplitude.

This algorithm uses a human factor to help determine thresholds. The leading source of fault in this Pan and Tompkins technique could be the operator's experience in setting thresholds.

#### 6.1.2. Hilbert Transform (HT)

As a result of the physiological state, all physiological signals are nonlinear and nonstationary. The Hilbert transform is the finest technique for analyzing signals that do not typically trail an even arrangement or stay stagnant (HT). All of the limitations of FFT and DWT are overcome by HT.

The first signal is decomposed into intrinsic mode function (IMF) and then the Hilbert transform is used to convert this IMF into frequency domain signal. It is defined as the phase angle shift of all components of a signal h(t) by 90^o^ in the Hilbert transform. With h(t) as its signal representation, the Hilbert transform of h(t) can be inscribed as

(4) $$\begin{array}{c} \hat{h}\left(t\right)=\frac{1}{\pi }\int_{-\infty }^{\infty }\frac{h\left(p\right)}{t-p}\text{d}p. \end{array}$$

Researchers in [13, 25–28] used HT as an implementation for ECG QRS recognition using the HT technique.

#### 6.1.3. Optimum Reduced Order Filter Design

As it can be perceived from the above equations that basic IIR filter requires higher order filter of 16 orders, in this paper MIN-MAX optimization is proposed to diminish the order of the transfer function. The numerator and denominator coefficient vectors of the IIR filter as [b1, a1] are optimizing Min-Max optimization.

I. Optimization problem: this paper formulates the blind min-max optimization problem for ECG peak detection. In the min-max optimization, the problem is to maximize inner and minimize outer objective function *f* (*x*_1_, *x*_2_) which can be mathematically given as

(5) $$\begin{array}{c} \;\underset{x1\in X}{\min}\underset{x2\in X}{\max}\;f\left(x_{1},x_{2}\right), \end{array}$$

where *x*_1_ and *x*_2_ are optimization variables, differentiable objective function is  *f*, and  *X* ⊂ *R*^*dx*_1_^, Y ⊂*R*^*dx*_2_^  are convex sets.

Transfer function coefficients are optimized sequentially as shown in sequential procedure for Min-Max optimization.

1. The long-term and short-term ECG peak detection samples are proposed to evaluate a specific case. Short-term alphabet ECG peak detection samples are recorded.
2. They are proposed to design optimization method for minimized order IIR filter denoising of herring aid signal.
3. Proposed IIR filter has to be deliberated by the pass band and stop band filter for denoising.
4. Adoptive amplitude and threshold scaling is proposed for short-term ECG peak detection.
5. It is also proposed to evaluate the FFT of the filtered responses for data preservation.
6. The transfer function comparison is used for evaluating the performance of filtering.

The transfer function of the condensed order optimum IIR filter corresponding to the previous shown 16 order IIR filter transfer functions is given as discussed below.

II. Transfer functions analysis: the transfer functions for different stages of the propose reduced order IIR filter design are presented in Table 1. It can be perceived that our method significantly minimizes the filter order and also simultaneously preserves the nature of ECG signal as already discussed previously. It can be observed that IIR filter is designed with 16 order and after optimization the reduced order filter has order of 2.

## 7. The Proposed Algorithm

All the steps followed in the proposed algorithm are mentioned below:

1. The ECG data having arrhythmia cases have 48 channels. 30 channels data are loaded as mat files for classification
2. Define actual array of ECG features
3. Set sampling frequency Fs (500 Hz) and standard QRS interval (0.099 sec.), i.e., QRS(t)
4. Baseline wondering is performed by using 60 order FIR high pass filter
5. Design an optimum 150 Hz IIR low pass filter
6. Design a pass band butter worth filter having lower and upper cutoff frequencies *F*_L_ and *F*_H._
7. Design a stop band Butterworth IIR filter with lower and upper cutoff frequencies *F*_L1_ and F_H1_
8. Apply min-max optimization over filter coefficients
9. Reduce the order of IIR filter
10. Remove power line interference with 100 coefficient FIR stop band filter
11. Plot and evaluate the filter coefficients
12. Implement the Hilbert transform on filtered ECG signal
13. Obtain QRS peak and the RR and QRS interval heart rate for peak detection and ECG signal feature extraction
14. Calculate the mean of regular heart rate and irregular heart rate
15. Calculate the database distances between regular and irregular data and apply threshold-based detection approach to detect regular and irregular ECG data

The proposed algorithm flow chart is as follows Figure 4.

## 8. Result and Description

In this paper, the prime concern is to demonstrate the performance improvement of ECG classification by using the optimized IIR filter design. The MIT-BIH Arrhythmia ECG bed database [7] is applied for the classification of the regular and irregular ECG data. Out of the 48 available channels of the humans, the 30 ECG data are selected for the current study, having the versatile range of the ECG data. The input ECG data are presented in Figure 5. These ECG data are recorded at the rate of the 360 samples per second. The description of MIT-BIH database used and the details of the cases considered in Figure 5 for study are shown in Table 2.

In Figure 5, (x)-axis denotes time in seconds and *y*-axis denotes amplitude. Figure 5 gives details plotting of database and we can observe that each input has different behavior.

Among all the 30 ECG channels, six ECG channels as 102, 106, 109, 200, 208, and 228 are selected with different features difficulties to represent the visual results for the peak detection algorithm. These ECG data are presented in Figures 6(a)–6(f). These channels have the most of the irregular variations in the ECG data. Thus, it becomes significant to demonstrate the efficient peak detection method over them. Another reason of selection of these channels is that they are also considered by many existing ECG peak detection methods as in [29].

In Figure 6, (x)-axis signifies the number of ECG samples and *y*-axis signifies amplitude of ECG signal.  Figure 6(a)-6(f) represents the waveform plot of channel number 102, 106, 109, 200, and 208 and channel number 228. From Figure 6 we can observe that 6(b), 6(d), and 6(f) present a good peak detection which can be used for ECG peak in peak detection. Moreover, Figures 6(a), 6(c), and 6(e) have peaks very close to each other.

### 8.1. Min-Max Optimization for Optimum Filter Design

When it comes to designing an optimal reduced order IIR filter, this paper proposes a primary modification to the process of ECG signal processing. Smoothening is achieved by replacing the conventional FIR low-pass filters with the proposed reduced order IIR filter design.

Figure 7 presents the sequential results for the ECG signal filtering using the proposed IIR filter with optimization techniques. It is clearly observed that band pass filter and the IIR filter stages do not clearly represent the *Q* and S peaks signals although the *R* peaks are preserved. But as our goal is to design the QRS interval based classification method; thus, it is proposed to improve the performance of the IIR filtering. Therefore, a min-max optimization is used for scheming the condensed order transfer function for ECG filtering. It is clear from the final row in Figure 7 that the projected approach considerably smoothens the artefacts and also preserves the features of the QRS peaks [22, 29]. It can also be perceived that the amplitude of the minimized order filter is also much better than the amplitude of the band-pass filter and IIR filter design. There are no negative values in the reduced order filtered signals. It is because min-max optimization eliminates the negative coefficients from transfer function, thus all the values are positive only. The amplitude range is cut down from the 800–1600 to the vicinity 300 to 600 m-volt.

### 8.2. Results of Hilbert Transforms

In this paper the preprocessing stage is followed through the Hilbert transform stage. The filtered ECG signal is passed to the Hilbert transform block in order to improve the efficiency of the peak detection method. The basic uses of the Hilbert transform (HT) is to improve the efficacy of the *R* peak recognition for envelop detection. The use of HT [18] usually shifts positive and negative frequency components by −90° and +90°, respectively; on the other hand, all the amplitudes of transform domain function F[x(t)] remains constant as the *R* peaks of the ECG. In this way, it is determined that the orthogonality of x(t) with respect to the harmonic conjugate xH(t) is established, which is harmonic conjugate of x(t).

The results of introducing the Hilbert transform over the filtered signal using the optimum reduced order filter design for three signals 104 m, 109 m, and 228 m are presented in Figures 8, 9, and 10 correspondingly. In Figures 8, 9, and 10, for the sake of clarity, portions of the filtered signal are shown as zoom version in the two columns of the same figure, respectively, for signals in column one. It is clear that using the Hilbert transform may improve the gain of the *Q*, R, and S lower peaks. Thus in turn it may improve the peak detection and also preserve the original ECG signal pattern.

### 8.3. Results of Filter Design

The visual representation of the result comparison for the proposed IIR filter design is shown in Figure 11. The figure presets the proposed ECG signal preprocessing results plotted for the full ECG length of samples.  Figure 11(a) represents the results for 100^th^ ECG data and Figure 11(b) represents results for of the 106^th^ ECG data, where *x*-axis signifies the number of samples taken and y-axis signifies the amplitude of ECG signal. The filtered data have three stages of the proposed IIR filter designs. The first stage is baseline wondering noise removal using band pass filter. Secondly, results are shown after stop band as IIR filter and finally results with min-max optimization for reduced order filter are represented in the figure. It can be observed that the proposed filter design enhances the magnitude of signal and also preserve the nature of the original ECG signal as there is no negative coefficient after the optimization.

Further analysis is much clear with the better representation of filtering for 3500 and 2000 initial samples shown in Figure 12 with clear view. The figure represented the results for the ECG 100m signal. The baseline filtering effects are clearly visible in Figure 12(b)) for 2000 samples as it gives zoomed view of filtering. Here in Figures 12(a) and 12(b) also *x*-axis characterizes the number of samples considered for experiment and *y*-axis characterizes amplitude of ECG signal.

From Figures 12(a) and 12(b), it can be easily concluded that baseline wandering is removed and the signal got smoothened after this filtering.

### 8.4. Results of QRS Peak Detection

This section presents the consequences of QRS peak recognition for the four input ECG signals in Figure 13. It can be observed that peaks are efficiently identified for *Q*, R, and S peaks for all four cases with the proposed method.

For QRS detection, we have considered ECG signal of channel no. 102m in Figure 13(a), channel no. 109m in Figure 13(b), channel no. 208m in Figure 13(c), and channel no. 228m in Figure 13(d). In these figures, x-axis characterizes number of samples and *y*-axis characterizes voltage of ECG signal for that particular channel. With the analysis of all these figures, we can conclude that filtering of the ECG signal peaks is efficiently detected which helps in *Q*, R, and S peaks accurate detection.

In the next section, we will discuss the evaluation of the proposed ECG signal classification.

### 8.5. Evaluation of Proposed ECG Classification

In this section, the paper compares the classification efficiency of the three different approaches of the QRS peak detection as standard Pan–Tompkins [17] method of 60 order FIR filter, and our proposed approach of optimum reduced order IIR filter. Our paper presented three different ECG classification rules. The rules of the HRV based ECG classifications, regular or irregular ECGs, are summarized in Algorithms 3, 4, and 5, respectively.

### 8.6. Parametric Evaluation of Classification

The major concern is to demonstrate the improvement in the classification efficiency with the proposed method. To calculate efficiency, we will calculate few parameters such as sensitivity, specificity, accuracy, and precision.

A false negative (Fn) is generated when the procedure is unable to identify an accurate beat. Fns are extracted from the MIT-BIH record's equivalent annotation case. A false positive (Fp) is an untrue beat outcome, where true positive (Tp) is the precise beat identified based on the procedure that has been proposed. Moreover, true negative (Tn) is correct not detected beats. These parameters are calculated by

(6) $$\begin{array}{c} \text{Tn}=\text{sum}\left(\text{Diff}==0\;\&\text{ Actual}==0\right); \end{array}$$

(7) $$\begin{array}{c} \text{Tp}=\text{sum}\left(\text{Diff}==0\;\&\text{ Actual}==1\right); \end{array}$$

(8) $$\begin{array}{c} \text{Fn}=\text{sum}\left(\text{Diff}∼=0\;\&\text{ Actual}==1\right); \end{array}$$

(9) $$\begin{array}{c} \text{Fp}=\text{sum}\left(\text{Diff}∼=0\;\&\text{ Actual}==0\right); \end{array}$$

Sensitivity: this refers to the percentage of exact beats that occur in a given recording session which were correctly identified by the algorithm and shown in the following equation:

(10) $$\begin{array}{c} \text{Sensitivity}=\frac{\text{Tp}}{\left(\text{Tp}+\text{Tn}\right)}*100. \end{array}$$

Specificity: the ability to correctly identify people who do not have a disease using a test. Specificity is shown in the following equation:

(11) $$\begin{array}{c} \text{Specificity}=\frac{\text{Tp}}{\left(\text{Tp}+\text{Fn}\right)}*100. \end{array}$$

Performance accuracy is the utmost instinctive enactment metric because it is a simple relationship of appropriately anticipated interpretations to all interpretations made.

Precision: it is defined as the number of correctly predicted positive observations divided by the total number of predicted positive observations. Accuracy and precision are mathematically represented as

(12) $$\begin{array}{c} \text{Accuracy}=\frac{\left(\text{Tp}+\text{Tn}\right)}{\left(\text{Tp}+\text{Tn}+\text{Fn}+\text{Fp}\right)}*100, \end{array}$$

(13) $$\begin{array}{c} \text{Precision}=\frac{\text{Tp}}{\left(\text{Tp}+\text{Fn}\right)}*100. \end{array}$$

In this article, we have evaluated Tn, Tp, Fn, and Fp by using different classification rules like Pan–Tompkins, FIR filter, the proposed methodology of QRS detection and the proposed methodology of fuzzy methods encapsulated in Table 3.

Moreover, precision, accuracy, specificity, and sensitivity parameters are evaluated by using different classification rules like Pan and Tompkins, FIR filter, the proposed methodology of QRS detection, and the proposed methodology of fuzzy methods encapsulated in Table 4.

Further, HRV rules are applied to check the classification of irregularity for all of the ECG signal channels from our database and compared with actual training data to check the efficiency of our proposed method.

From Table 5 we can conclude that the proposed fuzzy HRV rule based classification is very close to actual training data for irregularity detection.

### 8.7. Time Domain HRV Parameter Analysis

The analysis of time domains statistical HRV parameters are presented for the proposed ECG classification and peak detection method. Various parameters in time domain are calculated using the RR intervals used for analyzing the ECG signal. The parameters used for analysis in this paper are defined as follows:

(a) Standard deviation of NN interval (SDNN): the *R* to *R* time is calculated for each pair of RR interval. The SDNN is defined as the standard deviation (SD) of the RR intervals.
(b) Root mean square SD (RMSSD): the RMSSD value is calculated by mean square differences of the calculated approximate derivatives using RR interval, mathematically defined as
  (14) $$\begin{array}{c} \text{RMSSD}=\sqrt{\frac{1}{M}\left(\text{diff}{\left({\text{RR}}_{\text{Region}}\right)}^{2}\right),} \end{array}$$
  where *M* is the length of the RR interval vector represented as RR_Region_. .
(c) NN50 value: the NN50 value is defined as the number of *R* to *R* intervals greater than the 50 ms interval.

The statistical values of measured parameters are shown in Table 6 for six input ECG signals with the proposed method of peak detection.

From Table 6, we can conclude that SDNN is obtained maximum for 228m channel and minimum for 106m ECG channel. The parameter RMSSD is evaluated maximum for 102m ECG channel and minimum for 106m ECG channel. NN50 parameter is the highest for 200m ECG signal and the lowest for 109m ECG signal. The heart beat is evaluated maximum for 106m ECG channel and minimum for 106m ECG channel.

### 8.8. Nonlinear HRV Analysis

The analysis of Poincare architecture is a nonlinear geometric way to test the HRV dynamic nature. Poincare plots are a visual graphs where each RR interval is arranged as a function of the previous RR interval as shown in Figure 14. Poincare plots were assessed in a qualitative manner using their visual pattern when constructing the structure divided into functional categories that reflect that range of heart failure.

Plots can be evaluated extensively by calculating the SD indicators of the structure. The Poincare plot provides abstract details and detailed details of beat-to-beat nature of conduction of the heart. Poincare plotting can be the best way to monitor the dynamic change of self-care during anesthesia.

The value of each consecutive RR intervals pair is representing the point on the plot.

## 9. Conclusion

The QRS peak detection is having significant role for disease detection and identification of heart rate variability (HRV). The time history analysis plays impactful role for HRV detections. Therefore, this paper proposed to design a new approach of QRS peak detection and classification of the ECG data. The design of reduced order IIR filter is proposed for the low pass smoothening of the ECG signal data. The min-max optimization is used for optimizing the filter coefficient for designing the reduced order filter design. In addition, the ECG classification based on the HRV parameters is presented to demonstrate the efficiency of the proposed filter design. Three approaches of HRV-based classification are presented using the Pan–Tompkins [17] approach, using FIR filter of 60 order and the proposed filter design. In this paper, for performance improvement, a new fuzzy-based ECG classification rule is proposed. The rule takes the QRS interval, HRV distance measure, and the heart beats count into consideration to categorize the ECG data as regular or irregular. The proposed method uses the true actual training states of ECG data for indicating the classification efficiency of the projected filtering method. The proposed QRS peak detection and classification are simple and suitable to use for real time applications.

The 30 ECG Arrhythmia data from MIT-BIH is used for experimentation and classification. The proposed filter is combined with the Hilbert transform for *Q* and S peak detection. It is determined that the projected optimum filter enhances the amplitude and preserves the ECG nature, therefore improving the detection efficiency. The true positives are increased and false negatives are reduced with the use of the proposed classification rule. This paper presented the results of Poincare plots for ECG analysis. It can be determined that the use of the projected filter with optimization method outpaces since 100% precession is achieved and the accuracy is increased by around 13% over basic Pan–Tompkins method and around 8% over the existing FIR-filter-based classification rules. In the future, we would like to apply our analysis method to finding other peak spots in ECG signals. Detecting various forms of peaks in ECG signal can provide more valuable information for detecting CVDs and create a number of related applications.

## Figures and Tables

**Figure 1:** Two cycle regular ECG waveform.

**Figure 2:** Sequential processes of ECG peak detection and classification.

**Figure 3:** Two-stage basic IIR filter design process.

**Figure 4:** Flow chart of the proposed QRS peak detection and disease detection algorithm.

**Figure 5:** Input MIT-BIH/PhysioNet ECG Arrhythmia database of 30 persons recorded for over 30 min, 5.556 sec, used for the current study. These data are 100,101,102,103,104,105, 100, 101, 102, 103, 104, 105, 106, 107, 108, 109, 111, 113, 114, 200, 201, 202, 203, 207, 208, 209, 210, 212, 213, 214, 215, 217, 219, 221, 222, 228.

**Figure 6:** Six unique ECG data with different features difficulties are considered for perceptual result representation: (a) 102, (b) 106, (c) 109, (d) 200, (e) 208, and (f) 228.

**Figure 7:** An example of the sequential filtered ECG signal data with proposed optimum IIR filter design process. (a) Original ECG data 106. (b) Band pass filter output. (c) IIR filtered ECG data. (d) Filter data with optimum reduced order data using min-max optimization.

**Figure 8:** Results of the calculated Hilbert transform for increasing efficiency of R peak detection for channel no. 104.

**Figure 9:** Results of the calculated Hilbert transform for increasing efficiency of R peak detection for channel no. 109.

**Figure 10:** Results of the calculated Hilbert transform for increasing efficiency of R peak detection for channel no. 228.

**Figure 11:** The proposed ECG signal preprocessing plotted for the 3500 samples (a) 100^th^ ECG data and (b) of the 106^th^ ECG data.

**Figure 12:** Better representation of ECG signal artifact removal results shown for sample length of 2000 for the 100 m signal.

**Figure 13:** Results of the QRS peak detection for four ECG signals with the proposed optimum IIR filter method.

**Figure 14:** Results of the Poincare plot for HRV analysis of the six ECG signals. (a) For 102m.mat, (b) For 106m.mat, (c) For 109m.mat, (d) For 200m.mat, (e) For 208m.mat, and (f) For 228m.mat.

**Algorithm 1:** Pan–Tompkins.

**Algorithm 2:** FIRREGULAR filter.

**Algorithm 3:** Using QRS Interval.

**Algorithm 4:** Using QRS + HRV.

**Algorithm 5:** Fuzzy QRS + HRV.

**Table 1:** Transfer functions for different filters used for filter design of ECG peak detections.

Filter method	Designed transfer functions
FIR filter 60 order low pass filter	h_60 = -4.168e-19 s^60 + 0.0004528 s^59 0.0008864 s^58 + 0.001208 s^57–0.00127 s^56 + 0.0009014 s^55–5.451e-18 s^54–0.001371 s^53 + 0.002909 s^52–0.004086 s^51 + 0.004272 s^50–0.002955 s^49 + 3.791e-17 s^48 + 0.004159 s^47–0.008473 s^46 + 0.01146 s^45–0.01158 s^44 + 0.00778 s^43–2.215e-17 s^42–0.01052 s^41 + 0.02122 s^40–0.02865 s^39 + 0.02921 s^38–0.02005 s^37 + 2.962e-17 s^36 + 0.02986 s^35–0.06616 s^34 + 0.1037 s^33–0.1364 s^32 + 0.1587 s^31 + 0.8331 s^30 + 0.1587 s^29–0.1364 s^28 + 0.1037 s^27–0.06616 s^26 + 0.02986 s^25 + 2.962e-17 s^24–0.02005 s^23 + 0.02921 s^22–0.02865 s^21 + 0.02122 s^20–0.01052 s^19–2.215e-17 s^18 + 0.00778 s^17–0.01158 s^16 + 0.01146 s^15–0.008473 s^14 + 0.004159 s^13 + 3.791e-17 s^12–0.002955 s^11 + 0.004272 s^10–0.004086 s^9 + 0.002909 s^8–0.001371 s^7–5.451e-18 s^6 + 0.0009014 s^5–0.00127 s^4 + 0.001208 s^3–0.0008864 s^2 + 0.0004528 s - 4.168e-19

Pan–Tompkins 32 order LPF	*h*_32_=(0.03125 *s*^12^ − 0.0625 *s*^6^+ 0.03125)/*s*^2^ − 2 *s* + 1

Band pass filter	*h*_1_=( 0.2066 *s*^4^ − 0.4131 *s*^2^+ 0.2066)/*s*^4^+ 0.5488 *s*^3^+0.4535 *s*^2^+ 0.1763 *s* + 0.1958

IIR filter 16 order	$h_{2}=\begin{array}{c} 0.32\;s^{16}+4.517\;s^{15}+30.45\;s^{14}+130\;s^{13}+393.2\;s^{12}+\;\\ 892.9\;s^{11}+1574\;s^{10}+2196\;s^{9}+2452\;s^{8}+2196\;s^{7}+1574\;s^{6}\\ +\;892.9\;s^{5}\;+393.2\;s^{4}+130\;s^{3}+30.45\;s^{2}+4.517\;s\;+\;0.320 \end{array}/\begin{array}{c} s^{16}+12.12\;s^{15}+70.25\;s^{14}+258.1\;s^{13}+672.2\;s^{12}\\ +1316\;s^{11}+2004\;s^{10}+2419\;s^{9}+2340\;s^{8}+1819\;s^{7}+113\;s^{6}\;\\ +559.4\;s^{5}+214.8\;s^{4}+62\;s^{3}+12.7\;s^{2}+1.649\;s\;+0.102 \end{array}$

Optimum reduced order IIR filter	*h*_opt_=(3*s*+14)/41

**Table 2:** Description of MIT-BIH database used for the study.

	Data from samples numbered as											
Futures	100	101	102	103	104	105	106	107	108	109	111	113
Beats	2273	1865	2187	2084	2229	2572	2027	2173	1774	2532	2124	1795
Gender	M	F	F	M	F	F	F	M	F	M	F	F
Age	69	75	84	—	66	73	24	63	87	64	47	24

*Data from samples numbered as*												
Futures	114	200	201	202	203	207	208	209	210	212	213	214
Beats	1879	2601	2000	2273	1865	2187	2084	3005	2650	2748	3251	2262
Gender	F	M	M	M	F	F	M	M	M	F	M	M
Age	72	64	68	69	75	84	-	62	89	32	61	53

*Data from samples numbered as*												
Futures	215	217	219	221	222	228	215					
Beats	3363	2208	2287	2427	2483	2053	3363					
Gender	M	M	M	M	F	F	M					
Age	81	65	—	83	84	80	81					

**Table 3:** Comparison of parameters of different preprocessing approaches for different classification methods.

Classification rule	Tn	Tp	Fn	Fp
Pan–Tompkins [16]	5	152	2	8
FIR filter	6	16	7	1
Proposed_QRS_Dist	6	15	8	1
Proposed fuzzy	0	23	0	7

**Table 4:** Comparison of accuracy and precision for different preprocessing approaches for two different classification rules.

Classification rule	Precision	Specificity	Sensitivity	Accuracy
Pan–Tompkins [16]	65.2174	86	75	66.6667
FIR filter	69.5652	69.5652	72.7273	73.3333
Proposed_QRS_Dist	65.2174	65.2174	71.4286	70
Proposed fuzzy	100	100	100	76.667

**Table 5:** Result comparison of HRV rules for ECG signal classification for irregularity.

Records	Actual training data	Pan–Tompkins	With FIR filter	Proposed fuzzy HRV rule
100	Regular	Regular	Irregular	Regular
101	Irregular	Irregular	Irregular	Regular
102	Irregular	Irregular	Irregular	Regular
103	Regular	Irregular	Irregular	Regular
104	Irregular	Regular	Irregular	Regular
105	Regular	Regular	Regular	Regular
106	Regular	Irregular	Irregular	Regular
107	Irregular	Irregular	Irregular	Regular
108	Regular	Irregular	Irregular	Regular
109	Regular	Regular	Regular	Regular
111	Regular	Irregular	Irregular	Regular
113	Regular	Irregular	Irregular	Regular
114	Regular	Irregular	Regular	Regular
200	Regular	Regular	Regular	Regular
201	Regular	Regular	Regular	Regular
202	Irregular	Irregular	Regular	Irregular
203	Regular	Regular	Regular	Regular
207	Regular	Regular	Regular	Regular
208	Regular	Regular	Regular	Regular
209	Regular	Regular	Regular	Regular
210	Regular	Regular	Regular	Regular
212	Irregular	Regular	Regular	Regular
213	Regular	Irregular	Irregular	Regular
214	Regular	Regular	Regular	Regular
215	Irregular	Irregular	Irregular	Regular
217	Regular	Irregular	Irregular	Regular
219	Regular	Regular	Regular	Regular
221	Regular	Regular	Regular	Regular
222	Regular	Regular	Regular	Regular
228	Regular	Regular	Regular	Regular

**Table 6:** Statistical values of measured parameters for HRV analysis.

ECG signals parameters	ECG 102m	ECG 106m	ECG 109m	ECG 200m	ECG 208m	ECG 228m
SDNN	80.3078	9.1564	35.4786	13.82	42.2744	49.3268
RMSSD	104.9028	9.9598	20.0403	12.6611	55.5034	66.5002
NN50	76	70	67	85	82	70
Heart beats	0.0099	0.0106	0.0079	0.0085	0.0092	0.0096

## Data Availability

The data underlying this article are derived from online sources in the public domain as PhysioNet. These heart rates (ECG) are measured over 3 R-R intervals in beats per minute and available at https://physionet.org/physiobank/database/html/mitdbdir/records.htm.
